This article has been retracted.

# Noscapine, an Emerging Medication for Different Diseases: A Mechanistic Review

**DOI:** 10.1155/2021/8402517

**Published:** 2021-11-29

**Authors:** Pouria Rahmanian-Devin, Vafa Baradaran Rahimi, Mahmoud Reza Jaafari, Shiva Golmohammadzadeh, Zahra Sanei-far, Vahid Reza Askari

**Affiliations:** ^1^Department of Pharmaceutics, School of Pharmacy, Mashhad University of Medical Sciences, Mashhad, Iran; ^2^Department of Cardiovascular Diseases, Faculty of Medicine, Mashhad University of Medical Sciences, Mashhad, Iran; ^3^Nanotechnology Research Center, Pharmaceutical Technology Institute, Mashhad University of Medical Sciences, Mashhad, Iran; ^4^Department of Pharmaceutical Nanotechnology, School of Pharmacy, Mashhad University of Medical Sciences, Mashhad, Iran; ^5^Applied Biomedical Research Center, Mashhad University of Medical Sciences, Mashhad, Iran; ^6^Department of Pharmaceutical Sciences in Persian Medicine, School of Persian and Complementary Medicine, Mashhad University of Medical Sciences, Mashhad, Iran; ^7^Department of Persian Medicine, School of Persian and Complementary Medicine, Mashhad University of Medical Sciences, Mashhad, Iran

## Abstract

Noscapine is a benzylisoquinoline alkaloid isolated from poppy extract, used as an antitussive since the 1950s, and has no addictive or euphoric effects. Various studies have shown that noscapine has excellent anti-inflammatory effects and potentiates the antioxidant defences by inhibiting nitric oxide (NO) metabolites and reactive oxygen species (ROS) levels and increasing total glutathione (GSH). Furthermore, noscapine has indicated antiangiogenic and antimetastatic effects. Noscapine induces apoptosis in many cancerous cell types and provides favourable antitumour activities and inhibitory cell proliferation in solid tumours, even drug-resistant strains, via mitochondrial pathways. Moreover, this compound attenuates the dynamic properties of microtubules and arrests the cell cycle in the G2/M phase. Noscapine can reduce endothelial cell migration in the brain by inhibiting endothelial cell activator interleukin 8 (IL-8). In fact, this study aimed to elaborate on the possible mechanisms of noscapine against different disorders.

## 1. Introduction

With the chemical formula C_22_H_23_NO_7_, noscapine is a benzylisoquinoline alkaloid compound found in Papaveraceae, Berberidaceae, and Ranunculaceae [1]. Although noscapine is extracted from alkaloid-rich plants, such as papaverine, it has none to mild effects on central nervous system (CNS) activities and does not cause respiratory suppression, euphoric, or addictive effects [2]. Initially, noscapine was considered and used clinically for its antitussive effects [3] and has shown minimal toxic effects in animals and humans [4]. Due to the lack of opioid effects, noscapine is a safe alternative to codeine and dextromethorphan for treating cough. Likewise, in the Netherlands, noscapine is considered the first-choice medicine for treating paediatric cough [5].

In the recent decade, various pharmacological properties have been expressed for noscapine, including inducing apoptosis in cancer cell lines and inhibiting tumour cell growth [6]. It has also been observed that noscapine can inhibit the bradykinin receptors in both *in vitro* and *in vivo* experiments [7, 8]. Furthermore, noscapine derivatives are structurally similar to colchicine in that both contain a dimethoxy phenyl group, which can act on its receptors and have similar effects to colchicine. Also, studies show that noscapine and its derivatives reduce the dynamics of microtubules by increasing the stopping time of microtubules [9]. Clinically, lack of systemic and histological toxicity, favourable oral bioavailability and pharmacokinetics (clearance about 10 hours), and appropriate tumour-targeting activities are deliberated good characteristics of noscapine [10]. Therefore, this study aimed to review the biopharmacy and pharmacokinetics anti-inflammatory, antioxidant, and anticancer effects of noscapine by focusing on its receptors and signalling pathways.

## 2. Methods

Scientific databases, including Web of Science, PubMed, Scopus, and Google Scholar, were searched in English until the end of July 2021. The search terms were critical words, including “immunomodulation”, “anti-inflammatory” OR “immune system” OR “inflammation” OR “cancer” OR “tumour” OR “oxidative stress” OR “P-glycoprotein (P-gp)” OR “cell toxicity” OR “anti-mitotic”, OR “benzylisoquinoline alkaloid” AND “noscapine”, “Opiate”, “Papaveraceae”, and their combinations. All *in vitro* and *in vivo* studies and clinical trials examining the biopharmacy and pharmacokinetics anti-inflammatory and anticancer effects of noscapine were included. Unpublished data, “letters to the editor”, and non-English articles were also excluded. We have reviewed about 472 research articles, and finally, the results of 67 articles were evaluated and scrutinised for the present review study.

## 3. Results

### 3.1. Biopharmacy and Pharmacokinetics of Noscapine

#### 3.1.1. Physical and Chemical Characteristics

After morphine, noscapine is the most abundant alkaloid in the *Papaver somniferum* [11]. The French chemist Charles Derosne isolated noscapine from opium in 1803 and named it “sel narcotique de Derosne” [1]. Noscapine has a molecular weight of 413.42 g/mol, and its molecular formula is C_22_H_23_NO_7_. It is a polar molecule with a melting point of 176°C and 1.395 g/mL density. It is a white powder that has a bitter taste and is odourless. Noscapine is almost insoluble in water (0.181 mg/ml), most soluble in vegetable oils (Log *P*=2.58), slightly soluble in alcohol and ether, and soluble in benzene and acetone [1, 12]. However, noscapine hydrochloride is freely soluble in water and ethanol (∼750 g/ml) [12]. In addition, noscapine has a stable metabolite called meconin, which is excreted in the urine and dissolves in water at an amount of 2.5 mg/mL at 25°C. This metabolite is a skin irritant [1]. Noscapine can cross the blood-brain barrier very quickly due to its high lipophilic properties [1, 12].

#### 3.1.2. Pharmacokinetics in Experimental Animals

In mice pharmacokinetics models, noscapine was administrated intravenous bolus at 10 mg/kg and orally at 75, 150, and 300 mg/kg and then extracted from the plasma by the protein-precipitation method [13]. Following 10 mg/kg intravenous dose, the average plasma concentration of 7.88 *μ*g/ml within 5 minutes after injection and declined with undetectable levels at 4 h. The mean of total body clearance and mean volume of distribution (V (d)) were 4.78 L/h and 5.05 l, respectively. Using the noncompartmental analysis, the mean area under the plasma concentration-time curve (AUC) for noscapine was 53.42, 64.08, and 198.35 h *μ*g/mL reaching maximum plasma concentrations (C (max)) of 12.74, 23.24, and 46.73 *μ*g/mL at a *t* (max) of 1.12, 1.50, and 0.46 h at the linearly increasing dose levels [13].

#### 3.1.3. Pharmacokinetics in Human

In humans, it has been shown that oral administration of 50 mg noscapine results in rapid absorption and a plasma concentration of 182 ng/mL, one hour after administration. Following the absorption, noscapine levels are reduced by 30%, with a half-life of 124 minutes and an absolute oral bioavailability [14]. Four hours after administering noscapine, its blood concentration level is undetectable, indicating an average total body clearance of 4.78 L/h with an average distribution volume of 5.05 L.

#### 3.1.4. Side Effects of Noscapine

A study in 1961 on cancer patients reported that 80% of patients showed no side effects when taking daily doses of up to 3 g/day, while the remaining 20% felt drowsy and pain in the belly. However, administration of 4–6 grams orally daily may cause headache, dizziness, and even coma [11, 15].

### 3.2. Anti-Inflammatory Effects

Inflammation is a complex process that protects tissues against various injuries in a particular way and is a controlled outcome between inflammatory and anti-inflammatory agents. Chronic inflammation occurs when the inflammation goes out of physiological condition. These conditions are seen in some diseases such as metabolic syndrome, rheumatoid arthritis, psoriasis, osteoarthritis, and cancer [16–20]. Eventually, chronic inflammation causes inflammatory disorders and pain through the secretion of inflammatory mediators, including prostaglandins, nitric oxide (NO), interferon *γ* (IFN-*γ*), and histamine [21].

Interestingly, various studies have indicated that noscapine has anti-inflammatory effects and significantly reduces the levels of proinflammatory factors such as interleukin 1*β* (IL-1*β*), IFN-*γ*, and IL-6. In this regard, in another study, Khakpour et al. examined the effect of noscapine against carrageenan-induced inflammation in rats. They found that noscapine at a dose of 5 mg/kg body weight in three hours after the injection has the most anti-inflammatory effects. Moreover, they showed that the amount of inflammation reduction at this dose of noscapine is approximately equal to the indomethacin as a known and standard anti-inflammatory medication [22, 23]. Furthermore, Shiri et al. concluded that noscapine prevented the progression of bradykinin-induced inflammation in the rat's foot by antagonising bradykinin receptors [22].

In addition, Zughaier et al. evaluated the anti-inflammatory effects of brominated noscapine. The brominated form of noscapine has been shown to inhibit the secretion of the cytokine TNF-*α* and the chemokine IP-10/CXCL10 from macrophages, thereby reducing inflammation without affecting macrophage survival [24]. Furthermore, the bromated derivative of noscapine has about 5 to 40 times more potent effects than noscapine [25]. Again, this brominated derivative also inhibits toll-like receptor (TLR), tumour necrosis factor *α* (TNF-*α*), and NO in human and mouse macrophages without causing toxicity [26]. Furthermore, brominated noscapine has potent anti-inflammatory activity in models of septic inflammation, inhibits inflammatory factors in a dose-dependent manner, and prevents the release of TNF-*α* and NO in human and mouse macrophages [27].

Another study on inflammatory bowel disease (ulcerative colitis) and colon cancer found that noscapine had an excellent anti-inflammatory effect that could significantly decrease the levels of proinflammatory factors such as IL-1*β*, IFN-*γ*, and IL-6, compared to the control group [26]. Additionally, it has been found that chitosan nanoparticles containing brominated noscapine derivatives could reduce proinflammatory cytokines such as IL-1*β*, IFN-*γ*, and IL-6 and inflammation within colon mucosal tissue [26].

### 3.3. Anticancer Effects

Studies have shown that noscapine inhibits cell proliferation in many cancer cells, even many drug-resistant strains, and does not affect healthy cells. Compounds that have inhibitory effects on microtubules activate the mitosis phase control station and arrest the cell cycle, thus maintaining the balance between the monomer and the tubulin polymer, the tubulin polymerising more than usual. Various studies have shown that noscapine has an inhibitory effect on the skin, ovarian, blood, breast, and glioblastoma cancers without causing dose-dependent toxicity to the tissues of the kidney, heart, liver, bone marrow, spleen, and small intestine [1].

Collectively, two mechanisms for effects of noscapine anticancer are suggested, including downregulation of HIF-1 (hypoxia-inducible factor-1) and VEGF expression [28, 29], which are essential for the formation of blood vessels [30]. The secondary mechanism is also antimitotic effects by its inhibitory effects on microtubules [31]. However, relatively high doses of noscapine (ED50 = 300 mg/kg) are necessary to induce anticancer activity [32].

Antimitotic effects of noscapine provide it as an attractive anticancer medicine or lead compound for many researchers [31]. However, noscapine targets microtubules and destabilises their dynamics. While it does not alter the microtubule arrangement of healthy cells, mammalian cells are disrupted during the mitotic phase of cell division, leading to programmed cell death [33]. In addition, although other drugs, such as colchicine and paclitaxel, also affect tubulin, noscapine binds to different sites of tubulin due to structural differences from other medications [34]. Due to its antimitotic effects, noscapine has been found in various cancers such as lymphoma, melanoma, breast, ovarian, and bladder cancers [31]. Quisbert-Valenzuela et al. showed that noscapine has a selective apoptotic effect on different breast cancer cell lines, attributed to the inactivation of NF-*κβ* and activates apoptotic pathways [35].

#### 3.3.1. Breast Cancer

For example, Chougule et al. [36] found that noscapine exerts its antitumor effect in a dose-dependent manner. Therefore, they applied an oral dose of 550 mg/kg of noscapine alone and oral administration of 300 mg/kg/day combined with intravenous administration of doxorubicin (DOX, 1.5 mg/kg) on the MDA-MB-231 breast cancer tumours xenograft model [36]. It has been observed that administration of low concentrations of noscapine has improved the antitumor activity of DOX by three times in triple-negative breast cancer. In an additional experiment, noscapine with a concentration of approximately 36 *μ*M (IC50 = 36 *µ*M) can inhibit the proliferation of breast cancer cells [36].

A noscapine derivative called NPN (VinPhe-Nos) has great potential in treating invasive cancers by severely inhibiting new colonies and arresting the cell cycle in the G2/M phase and the S phase [37, 38]. In addition, studies have shown that the noscapine NPN derivatives can bind to tubulins and disrupt the tertiary structure of the protein [39]. This study also showed that NPN structurally altered tubulin protein and increased colchicine binding to tubulin [39]. Noscapine causes only minor damage to cell microtubules, but NPN severely damages microtubules, altering their arrangement and preventing them from rearranging [40].

#### 3.3.2. Lung Cancer

In one study, it has been demonstrated that the combination of noscapine 300 mg/kg/day orally and gemcitabine (30 mg/kg) inhibited lung tumour growth by an 82.9% rate. However, using each treatment, gemcitabine and noscapine alone could inhibit the tumour growth of non-small-cell lung cancer cells by 39.4% and 34.2%, respectively [32]. Thus, it indicates the synergism effect of noscapine on gemcitabine against non-small-cell lung cancer.

#### 3.3.3. Glioblastoma

Temozolomide (TMZ) is a chemotherapeutic agent used for glioblastoma that works by alkylating DNA and targeting proliferation [30]. Resistance to temozolomide involves several mechanisms, including the high activity of DNA-repairing enzyme (methylguanine methyltransferase) (MGMT) and the broad expression of antiapoptotic proteins and P-glycoprotein (P-gp) pumps [30].

Interestingly, it has been reported that noscapine alone could inhibit the proliferation of temozolomide-resistant glioblastoma cell lines [30]. However, studies show that the concentration of noscapine required to inhibit the growth of temozolomide-resistant glioblastoma cells, which is not very high (20–75 *µ*M) [41], but noscapine has significantly increased animal survival [30]. In addition, combination therapy of noscapine with temozolomide and cisplatin in xenografts significantly increased the efficacy of these drugs without showing any particular toxicity. Moreover, this *in vitro* combination therapy reduced cell proliferation and increased apoptosis in a tumour [41].

Although noscapine has low toxicity and desirable properties, it requires higher doses for providing anticancer effects, preventing noscapine from progressing in the pharmaceutical market. Numerous formulations have been developed, such as the preparation of nanoparticles [4, 42] and the water-soluble complex [43], but research is ongoing to address its pharmacokinetic limitations. The slow-release formulation of noscapine can provide a good plasma concentration of noscapine over a more extended period, which can help treat cancer [44].

In one study, the effect of noscapine solidified lipid nanoparticles on glioblastoma cells was investigated. The size obtained (101 ± 4.8 nm) for noscapine nanoparticles could be suitable for accumulation in tumour tissue by increasing penetration into the tissue and more lasting effects within the tissue [45]. In addition, these nanoparticles reduced side effects. However, it has been found that the cytotoxicity of noscapine IC50 nanoparticles is significantly higher than noscapine hydrochloride. In contrast, PEGylated lipid nanoparticles containing noscapine IC50 have less cytotoxicity than the free form of noscapine [46]. Furthermore, an examination of noscapine-containing PEGylated gelatin nanoparticles on glioblastoma cells showed that noscapine hydrochloride provided less cytotoxicity in the breast cancer cell line [47].

#### 3.3.4. Ovarian Cancer

A noscapine derivative called 9-nitro-noscapine has the effect of selectively binding to the ovulation of human ovarian cancer cells and human lymphoblastoid cells while not affecting the normal human cell cycle [48].

#### 3.3.5. Colon Cancer

A study also found that noscapine activated PI3K/mTOR signalling and reduced PTEN expression in LOVO 5FU and HT29/5FU cancer cells. In addition, it was found that noscapine significantly induces apoptosis of human colon cancer cells HT29/5FU and LOVO/5FU, indicating that it acts as an anticancer agent for treating colon cancer [49, 50].

The mechanism of drug resistance of cancer cells is that enzymes that directly regulate glycolysis and phenotypes are effective in drug resistance. Therefore, targeting critical metabolic enzymes can have a therapeutic effect by increasing drug-induced apoptosis in cancer cells [51]. According to the results, inhibition of the Warburg effect may increase the sensitivity of HT29/5FU and LOVO/5FU cells to noscapine. Therefore, it is estimated that targeting the development of Warburg improves the response to cancer cell therapy, and the combination of targeted drugs with inhibitors of cellular metabolism may be a promising strategy to enhance drug resistance in cancer.

#### 3.3.6. Osteosarcoma

One of the critical steps in cancer invasion and metastasis is the destruction of the extracellular matrix. MMP2 plays an essential role in the destruction of the extracellular matrix [52]. Noscapine in MG63 cells causes downregulation of MMP2 and simultaneously inhibits the EGFR pathway [53].

## 4. Targets of Noscapine, Receptors, and Signalling Pathways

### 4.1. Effects of Noscapine on Autophagy

Autophagy is a known cell pathway that removes macromolecules and destroys defective cytoplasmic components. According to previous studies, autophagy is directly related to vacuolation in the cytoplasm and the rearrangement of microtubule light-chain proteins. The rearrangement of microtubule light-chain proteins plays a role in the structure of autophagic vesicles. Recent reports indicated that autophagy is directly involved in controlling inflammatory responses [54]. Noscapine analogues significantly induced autophagy when in contact with macrophages. In fact, it has been observed in a study that inhibition of autophagy by 3-methyladenine (3-MA) reduced the anti-inflammatory activity of noscapine analogues. Thus, induction of autophagy, to some extent, is associated with the anti-inflammatory activity of noscapine and its derivatives [24]. It possibly interferes with the depletion of cytosolic signals by reducing the dynamics of microtubules, thereby reducing inflammatory responses.

Various studies have shown that ROS is also involved in the development of autophagy [55]. However, the relationship between apoptosis and autophagy is complex. Under certain conditions, autophagy selects adaptation to stress and prevents cell death. In other cases, autophagy is an alternative pathway to cell death. This evidence suggests that noscapine and its derivatives have anti-inflammatory activity without toxic effects on the cell. Furthermore, noscapine and its derivatives inhibit the transmission of cellular signals or delay transcription through proteins by acting on tubulin and reducing their dynamics [24].

### 4.2. Effects of Noscapine on PTEN Tumour Suppressors

PTEN tumour suppressors have been observed frequently in many human cancers, including mutated colon cancer. In particular, dephosphorylation of 3-phosphate catalyses the Inositol ring in PTP3, thereby inhibiting PIP2 bisphosphate, and inhibiting PI3K phosphorylation, thereby inhibiting AKT and kinase activity, leading to apoptosis [56]. Conversely, shutting down PTEN activates the PI3K/AKT signalling pathway, resulting in tumorigenesis [57].

Studies have shown that PTEN expression is induced in HT29/5FU and LOVO/5FU cells. Noscapine and PTEN interference with PI3K/mTOR activation reverses the effect of noscapine on cell apoptosis. Conversely, mutation of the PTEN gene can lead to abnormal PIP3 activation and prevent cell death. According to previous studies, P-expression PI3K and PmTOR were significantly increased in noscapine-treated HT29/5FU and LOVO/5FU cells after transfection with si-PTEN. Eventually, noscapine regulates mitochondrial damage, and the Warburg effect via PTEN induces apoptosis of colorectal cancer cells HT29/5FU and LOVO/5FU, and this mechanism is closely related to the PI3K/mTOR signal (Table 1) [56].

### 4.3. Effects of Noscapine on Bradykinin Receptors

The kinin system is one of the plasma protein systems involved in causing inflammatory reactions.

Bradykinin (BK), as the essential product of this system, along with other inflammatory mediators, including eicosanoids, histamine, oxygen-free radicals, and substance P, initiates inflammatory reactions, the activity of neurons in the pain pathway, and the onset of oedema in the affected area and damaging the blood-brain barrier [58–60].

Bradykinin is also responsible for the vasodilation caused by nitric oxide in smooth muscle [61].

The kallikrein-kinin system (KKS) is activated during inflammatory processes. Bradykinin (BK), calidin (Lys-BK), and their C-terminal metabolites increase vascular permeability, vasodilation, and expression of proinflammatory cytokines [61]. These effects are mediated by two receptors: the bradykinin B1 receptor and the B2 receptor. Usually, the B1 receptor is not present in healthy tissue; however, it is produced by tissue damage and proinflammatory cytokines through NF-*κ*B activation. Activation of B1 receptors increases vascular permeability, leukocyte adhesion, and expression of proinflammatory molecules such as vascular endothelial growth factor A (VEGF-A), VEGF-R2, ICAM-1, VCAM1, COX-2, and IL-1*β* in the diabetic retina [58–60].

Additionally, the BK induces angiogenesis by regulating basal FGF regulation (bFGF) through B1 receptors and by stimulating VEGF formation through B2 receptors in an absent vascular model. B1 receptors enhance compensatory angiogenesis in mouse models of obstructive vascular disease, and activation of these receptors also promotes the proliferation and survival of endothelial cells, while B1 receptor antagonists induce apoptosis [62].

#### 4.3.1. Ischemic Injuries

In ischemic injury of various organs, bradykinin B1 and B2 receptors are affected [58]. B2 receptors are expressed in the nervous system, while B1 is induced in response to inflammatory cytokines [63]. Activation of B2 receptors generates free radicals following ischemic damage in rats and impairs brain function [63].

Noscapine noncompetitively antagonises bradykinin receptors, crosses the blood-brain barrier easily, and targets the ischemic region of the brain for damage due to its protective and anti-inflammatory to reduce effects nervousness [8, 64]. Cytotoxic free radicals and released neurotransmitters, such as bradykinin, are involved in the pathogenesis of ischemic brain injury [65].

As a noncompetitive antagonist of bradykinin receptors, noscapine has been shown to protect against brain damage by reducing oedema against hypoxia/ischemia in neonatal mice. Also, it reduces damage to muscle activity [66]. Also, noscapine reduces cell death through various mechanisms, including inhibition of oxidative stress and reduced neutrophil permeability. It also reduces the permeability of vascular endothelium to nerve damage [58]. In addition, it increases reperfusion to the area of ischemic injury [8].

In a clinical study, oral administration of noscapine (50 mg/day for five days) to patients (hypoxic-ischemic) improves the clinical prognosis and significantly reduces mortality [67]. Moreover, in another clinical trial, oral administration of noscapine improved prognosis and reduced mortality in stroke patients, but the exact mechanism of action is still unclear [8].

Bradykinin receptor antagonists show protective effects in various tissue ischemia/reperfusion injury models, especially in the brain and kidneys [68].

#### 4.3.2. Cough

Noscapine has been shown to suppress cough induced by enalapril and FR19099F (a nonpeptide B2 receptor agonist) in guinea pigs, whereas it was not improved with naloxone premedication (a specific opioid antagonist) [69]. The findings showed that opioid receptors do not mediate the antitussive effects of noscapine. Accumulation of bradykinin has been suggested as an essential mechanism of cough induction by angiotensin-converting enzyme (ACE) inhibitors [70]. Mooraki et al., in 90% of patients with hypertension, stated that noscapine could suppress the cough caused by ACE inhibitors. Interestingly, some of these patients received lower doses of antihypertensive drugs with noscapine [7].

### 4.4. Effects of Noscapine on Tubulin

Drugs that act on microtubules, such as taxol derivatives and vinca alkaloids, are powerful anticancer drugs used in various cancers. However, these drugs are expensive to use due to limitations such as low solubility. Also, due to their nonselective action, these drugs have toxicities such as peripheral neuropathy, gastrointestinal toxicity, myelosuppression, and immune suppression [25]. Nevertheless, the FDA approved taxols in 1996 for breast and ovarian cancer [71]. The efficacy of taxol in treating invasive breast and ovarian cancer is an incentive to identify newer compounds that target microtubules but are less toxic than these compounds.

New compounds that target microtubules must have desirable properties, such as high water solubility, the ability to be taken orally, and the establishment of appropriate blood concentrations after consumption. In addition, these compounds can have a synergistic effect on the common drugs used in low amounts like taxols.

Noscapine is one of the compounds that is rapidly absorbed orally by the body and affects tubulin [14]. Noscapine binds to tubulin and disrupts the cell cycle by disrupting the ability of microtubules to accumulate. However, unlike most antitubulin agents, noscapine does not significantly alter the polymer mass of microtubules and does not cause severe damage to microtubules [72]. Instead, noscapine works by making minor changes in the accumulation and dynamics of microtubules [40]. Dynamic polymerisation and depolymerisation of microtubules to form mitotic spindles are an essential step in cell proliferation. This feature modulates the dynamics of microtubules and prevents cancer cell mitosis. Thus, noscapine works differently from the current anticancer drugs such as taxols and vinca alkaloids. Noscapine does not alter the arrangement of microtubules but reduces the dynamics of microtubules to activate mitotic activation sites [14].

Noscapine has been shown to bind to tubulin and stop tubules in the G2/*M* stage of mitosis. Also, noscapine does not alter the polymer-to-monomer ratio, unlike existing microtubule drugs that overpolymerise or destroy microtubules (such as taxols and vinca alkaloids) [77]. Therefore, it does not cause any blood or nerve poisoning [73]. Noscapine derivatives bind to tubules with greater affinity; however, these derivatives prevent cell proliferation and induce apoptosis death in human cancer cells [74]. Noscapine and its derivatives have been predicted to bind to tubules *α* and *β* of heterodimers near the colchicine binding site. However, they do not interfere with the binding of colchicine to its location [75].

Moreover, noscapine and two taxols (paclitaxel and docetaxel) bind to tubulin at different sites [76]. Thus, noscapine binds to the *α* and *β* sites of tubulin, but the two taxols attach to the *b* site [77, 78]. In fact, it suggests that noscapine may have a synergistic effect on tubulin inhibitors.

Despite the relatively low toxicity of noscapine, the anticancer activity of noscapine has been reported in the micromolar range. As a result, studies were done on its structure to produce compounds with greater strength. Further investigation of the mechanisms of noscapine revealed that this alkaloid increases the acetylation pattern of microtubules. Acetylated microtubules generally do not show sufficient dynamics [79]. Noscapine NPN derivative severely disrupts the network of microtubules, prevents their reassembly, and decreases the dynamics of microtubules [79].

Oxidative stress and reactive oxygen species (ROS) can damage cell microtubules [80] and inhibit the reshrinkage of microtubules [81]. ROS is known to be a suitable agent that interferes with the dynamics of microtubules [82]. In particular, the structure of the *α*-*β* tubulin heterodimer is susceptible to oxidation by ROS due to a hefty number of Cys-amino acids [83]. The physiological level of ROS facilitates the natural polymerisation of tubulin. In contrast, the high level of ROS can inhibit the dynamics and arrangement of tubulin through the oxidation of thiol groups [84]. Studies have shown that noscapine NPN derivatives can increase ROS levels in cells. Tubulin regulates mitochondrial membrane potential by interacting with mitochondrial ducts [85]. Therefore, it causes mitochondrial dysfunction, which causes more ROS production. As a result, mitochondrial function is impaired [86]. Also, noscapine can prevent the release of inflammatory mediators by affecting the tubules and reducing the dynamics of microtubules [14].

Various studies have shown that noscapine at maximum concentrations (100 *μ*M) does not affect the polymerisation of microtubules while keeping the microtubules stationary for a longer time, which stops mitosis [14, 87]. Nevertheless, it causes cellular ageing, which develops the further process of cell death, such as autophagy or apoptosis.

### 4.5. Effects of Noscapine on Sigma Receptors

Sigma ligands perform a wide range of actions, including protecting neurons against oxidative stress and treating cerebral ischemia in various cell lines, such as retinal ganglion cells [88]. In addition, sigma receptors affect the function of glutamate receptors during nerve damage and inhibit nerve cell destruction [89]. However, this protective mechanism effect is yet apparent, and studies have shown that glutamate is a critical neurotransmitter in the process of ischemic injury. Excessive increase in glutamate through NMDA receptor activation leads to increased Ca^2+^ accumulation within the cell, finally leading to cell damage and cell death, thus playing an essential role in stroke progression. Although blocking NMDA receptors reduces nerve damage, it also inhibits many of its positive effects. Therefore, we must modulate the function of NMDA receptors to control nerve damage [90].

#### 4.5.1. Ischemic Condition

Noscapine exerts its effects by acting on sigma receptors, previously classified as opioid receptors, that can be used as therapeutic targets to reduce cell damages [91]. In the mice model, Kamei et al. [92] showed that noscapine dose-dependently acts as a sigma receptor agonist. These data suggest that noscapine has a protective role in ischemic conditions [92]. Lack of oxygen or glucose is a significant cause of ischemic brain damage. Therefore, activating sigma-1 receptors by noscapine may provide neuroprotective effects against hypoxia or glucose-induced cell damage [93]. The concentration of glutamate and aspartate are increased in these conditions. Thus, NMDA receptors are stimulated, and subsequently, the intracellular Ca^2+^ ion concentration changes. Excessive Ca^2+^ increased within neurons, and endothelial cells can activate Ca^2+^-dependent enzyme cascades that activate various NO isoforms. Therefore, after oxygen or glucose deficiency or nerve damage, the NO level inside the cell increases (Figure 1) [94].

Proteolysis and production of reactive oxygen species cause cell death [95]. An essential mechanism of sigma-1 ligands is the modulation of intracellular calcium homeostasis and inhibition of ion channel function, thereby preventing damage caused by stimulation of glutamate receptors [96, 97]. They protect and reduce intracellular Ca^2+^ concentration [96, 97]. It has been shown that the intracellular level of Ca^2+^ is significantly increased in conditions of hypoxia or glucose deficiency or damages [93, 98]. However, treatment with noscapine 2 *μ*M prevents intracellular Ca^2+^ levels under hypoxia or glucose-deficient conditions [93, 98]. In fact, it has been shown that the protections were made by sigma-1 receptors, which blocks the receptors by BD-1047, a selective sigma-1 receptor antagonist; the protection will be hidden [93]. In this regard, Mueller et al. [99] showed that sigma-1 receptors exert neuroprotective effects on retinal ganglion cells by inhibiting Ca^2+^ signalling via VGCC type *L* [99].

Schulz et al. [100] showed that noscapine treatment decreased NO levels in H9C2 cells. In contrast, in the untreated group, NO levels in H9C2 cells increased significantly in response to OGD/R. It suggests that noscapine is a cardiac protective agent against NO damage. The results of this study showed that BD1047 increases NO levels in H9C2 cells, and noscapine significantly inhibits NO accumulation dose-dependently (4 *μ*M) [101]. Noscapine exerts its protective effect on the heart by binding to and activating the sigma-1 receptors, preventing necrosis and apoptosis in cardiomyocytes [100].

### 4.6. Effects of Noscapine on P-Glycoprotein (P-gp)

P-glycoproteins (P-gp) are the part of the membrane that binds to ATP. It is a transport protein and an active mediator that removes harmful substances to the cell (xenobiotic) from the cell. P-gp is overexpressed in cancer cells and reduces their sensitivity to various substances. One of the derivatives of P-gps is efflux mediators, which are still unknown [102]. The efficiency of this membrane transmitter requires a significant difference between the tendency to connect to the substrate site between the two media. Also, structural transitions are from very close junctions to the disintegration stages of an ATP hydrolytic process in the nucleotide-binding domain. In general, substrates for translocation tend to stimulate ATPase activity of P-gp, creating a solid bond between the binding site and the nucleotide-binding domains (NBDs) [103].

On the other hand, a group of compounds such as tariquidar have been shown to inhibit P-gp by inhibiting ATP hydrolysis [104]. Depending on its effect on ATPase, a compound can stimulate ATPase and act as a substrate, or it can act as an ATPase inhibitor and act as a P-gp inhibitor. Whether a compound has ATPase-stimulating or inhibitory activity depends on the conformation transition [105].

Noscapine has a modulating effect on efflux to be effective on resistant cancer cells by acting on P-gps. Noscapine modulates the activity of this protein by direct binding to P-gp [102]. Noscapine inhibits the proliferation and growth of cancer cells by reducing the substrate for P-gp transport. Noscapine and its derivatives are not substrates for P-gp but act as an inhibitor of this protein. The accumulation sites of P-gp-transported substrates are reduced by noscapine derivatives [106]. Noscapine affects resistant and sensitive cell lines, indicating that noscapine does not interfere much with P-gp [102].

Noscapine derivatives inhibit calcein-AM transport by P-gp in all cells. Therefore, compounds that alter ATPase activity can directly modify and inhibit P-gp function. The P-gp transfer mechanism requires the transfer of multiple structures and the interference of two different sites [107]. In particular, the displacement of the substrate involves the transfer from the connecting axis with a high inclination on the inside to a part with a slight tendency towards the outside of the cell. It is the active transfer that does this by consuming ATP [108].

Furthermore, it has been demonstrated that noscapine derivatives appear to affect P-gp expression in cells [109]. Also, the 9-nitro-noscapine derivative has been shown to induce apoptosis and stop mitosis in the ovaries and T-cells, which express P-gp, and are resistant to drugs such as paclitaxel and vinblastine [48]. Studies have shown that noscapine inhibits P-gp function through direct interaction with the P-gp transmitter [102].

### 4.7. Effects of Noscapine on VEGF

Angiogenesis is a vital phenomenon for the survival and development of solid tumours. In the absence of angiogenesis stimuli, tumours remain silent.

The essential precursors to angiogenesis in the body are vascular endothelial growth factor (VEGF), basal fibroblast growth factor (bFGF), and matrix metalloproteinase (MMP), and cyclooxygenase-2 (COX-2). Therefore, inhibiting angiogenesis requires antiangiogenesis factors or drugs that reduce the production of angiogenesis precursors, inhibit their function, or even prevent angiogenesis precursors from binding to their receptors.

Approximately 60% of malignant tumours have high concentrations of VEGF, so inhibiting the VEGF pathway is a way to control the rate of tumour growth. For example, treating patients with colon cancer with bevacizumab (a monoclonal antibody against VEGF) has improved patient survival [110, 111].

Tubulin-binding agents, such as taxanes, have been shown to have antiangiogenic effects [112].

Taxanes interfere with endothelial cell proliferation, migration, and differentiation into tiny capillaries to supply tumour food [113, 114]. As a result, taxanes have severe side effects, such as peripheral neuropathy, myelosuppression, alopecia, gastrointestinal toxicity, immune suppression, and cardiac toxicity [14, 115]. Recent studies show that noscapine has a similar anticancer activity to taxanes [29]. Noscapine downregulated hypoxia-mediated expression of HIF-1a in human glioma cells while reducing the potent cytokine secretion of VEGF. Also, high concentrations of noscapine inhibit tubule formation by human umbilical vein endothelial cells (HUVECS) [29].

Studies have shown that all noscapine derivatives showed dose-dependent antiangiogenic activity after 72 hours of treatment than those that did not receive noscapine [116]. According to the National Cancer Institute (NCI), IC 50 > 20, 6.9 *µ*M for Br-noscapine, and 6.79 *µ*M for folate-noscapine can inhibit VEGF (Table 2) [117]. In addition, studies have shown that all noscapine derivatives significantly prevent the formation of new blood vessels in endothelial cells [118].

It has been indicated in an *in vivo* study that a combination of noscapine and concomitant radiation therapy showed less cell proliferation, more apoptosis, and less angiogenesis and the formation of tubules in 2H11 endothelial cells compared with radiation therapy alone [29]. Thus, noscapine has anti-inflammatory, antiangiogenesis, and antimetastatic effects. In addition, examination of hypoxia conditions in human glioma cells has shown that noscapine has an inhibitory effect on VEGF, inhibits angiogenesis, and inhibits TNF-*α* and NF-*κ*B [116].

### 4.8. Effects of Noscapine on Apoptosis

Cell death occurs in two ways, including necrosis and apoptosis. Apoptosis, defined as programmed cell death, is an essential process that occurs during evolution, homeostasis, and disease. In addition, apoptosis plays a critical role in removing infected, damaged, or other unwanted cells from the body. Unlike necrosis or other cell death forms that arise from cell rupture, apoptosis is the silent immunological form of cell death that causes cells to rapidly phagocytosis and die without initiating an inflammatory process. Defects in apoptosis can play a role in developing diseases such as cancer, so one of the pathways studied in cancer is the path of apoptosis [119].

Apoptosis occurs due to the activation of caspase (cysteine-aspartic proteases) group enzymes. The intracellular ratio of apoptotic-inducing proteins (Bax) to antiapoptotic proteins (Bcl-2) determines the cell's susceptibility to apoptosis. Proapoptotic proteins (Bax) move from the cytoplasm to the mitochondrial wall, causing permeability of the outer mitochondrial wall, which leads to the release of cytochrome C and the onset of apoptosis [120].

Bax can create ion channels and holes in the membrane by modifying the mitochondrial membrane, releasing cytochrome C and apoptotic inducing factor (AIF) [121]. Bcl-2 is an inhibitor of apoptosis and affects the overall cascade of apoptosis by binding to Bax and BH3-only proteins like Bim. Phosphorylation of Bcl-2 by apoptosis signal-regulating kinase-1 reduces its binding to Bax and Bim, and thus its antiapoptotic activity is lost. The Bcl-2 family includes Bcl-2 and Bcl-X, which can inhibit apoptosis. Various studies have shown that these proteins inhibit apoptosis by inhibiting the release of caspases from mitochondria [122].

In a further study, Heidari et al. [123] represented that noscapine increased Bax/Bcl-2 expression ratio and induced apoptosis in both myeloid cell lines, apoptosis-resistant HL60 cells, and apoptosis-resistant K562 cells. However, the molecular mechanism of the anticancer effects of noscapine is unknown. In these noscapine-treated cells, caspases 2, 3, 6, 8, and 9 and poly(ADP ribose) polymerase activity increase, and the detection of phosphatidylserine in the outer layer of the cell membrane, chromatin nucleus, and fragmentation DNA induces apoptosis. Furthermore, noscapine increases Bax/Bcl-2 ratio by reducing Bcl-2 expression with Bcl-2 phosphorylation (Figure 2). In addition, this study showed that noscapine can induce apoptosis in leukemic cells resistant to apoptosis and could be a new candidate in treating blood malignancies (Table 2) [123].

Furthermore, in lung cancer cells, apoptosis is activated by the mitochondrial pathway after treatment with noscapine alone and in combination with cisplatin. This phenomenon is attributed to proapoptotic protein upregulation and antiapoptotic downregulation (Bcl-2) [124].

Newcomb et al. showed that noscapine (IC50 = 85–131 *µ*M) is a potent inhibitor of proliferation and induces apoptosis in human glioma. Stimulation of apoptosis is associated with activation of C-jun N terminal kinase (JNK) signalling, inhibition of extracellular regulated kinase (ERK) signalling, and phosphorylation of BCI-2 antiapoptotic protein. Noscapine induces apoptosis by secreting mitochondrial proteins, apoptosis-inducing factor (AIF), or cytochrome C. However, in some glioma cell lines, AIF release has been observed without cytochrome-C release (Figure 2). In fact, it suggests that noscapine induces apoptosis by AIF [87].

P53 is a tumour suppressor gene that is the most common cause of genetic alterations in human tumours. The product of this gene is a nuclear protein that is involved in cell cycle control, apoptosis, and deletion of gene stability. Thus, the function of the P53 protein usually is to regulate cell division—cell suicide, cell ageing, vascularisation, cell differentiation, and DNA metabolism. More than 26,000 genetic mutations have been reported for the p53 gene. The p53 protein is activated by N-terminus phosphorylation by the MAPK protein pathway and the ATM protein pathway. When p53 is phosphorylated, it loses its adhesion to MDM2. As a result, MDM2 protein binds to p53, blocks its action, and transfers it to the cell cytoplasm. Thus, P53 anticancer activity can be done in three ways: (1) P53 protein stimulates DNA repair proteins to address damage to genes. (2) P53 protein stimulates programmed death (when damaged cells are nonregenerating). (3) P53 protein maintains cell division in the S G1 phase to provide an opportunity for repair [125, 126].

Aneja and colleagues, in a study, claimed that noscapine, through the p53-dependent pathway, could inhibit cell growth and induce apoptosis in HCT116 colon cancer cells [49]. Because P53 is a significant regulator of apoptosis, expression of this factor in response to environmental stress by inhibiting microtubule dynamics can cause apoptosis in noscapine-treated cells. Noscapine leads to the accumulation of p53 within the cell, which in turn causes further secretion of p53. Thus, noscapine is p53-dependent and can induce apoptosis in cells by P21 [49].

### 4.9. Effects of Noscapine on Epidermal Growth Factor Receptor (EGFR)

Various studies have shown that by increasing gene expression and activating epidermal growth factor receptor (EGFR), many cellular processes such as cell proliferation, differentiation, migration, adhesion, protection against apoptosis, and angiogenesis are initiated, and the survival of breast cancer patients is reduced [127]. The structure of EGFR is tyrosine in nature and is involved in the activation of various pathways of AKT/PI_3_K (phosphoinositol tri-kinase) and RAF/RAS and MAPK. In addition, the EGFR-binding ligand activates the AKT/MAPK/STAT and PI3K/RAF/RAS signalling pathways, which together lead to proliferation, adhesion, and cell migration [128].

EGFR is a member of the ErbB family whose protein kinase activity is involved in the oncogenesis of several human cancers and is recognised as a therapeutic cancer target. EGFR on TYR 1068 also increases cyclin D1 expression and causes cell proliferation [53]. Noscapine has been shown to selectively inhibit EGFR phosphorylation on residual Tyr 1068, whose inhibition affects growth and attacks other cells [129]. In addition, EGFR aberrations affect various cellular signalling pathways in cancer cells, particularly PI3K/AKT and JAK/STAT [130].

Overexpression of EGFR is necessary to enhance motility and cell attack. *In vitro* data indicate that EGFR and AKT signalling play an essential role in the pathogenesis of osteosarcoma [131]. In one study, it has been represented that noscapine inhibited the migration and proliferation of MG63 osteosarcoma cancer cells in a concentration-dependent manner [53]. Moreover, it has been demonstrated that EGFR phosphorylation (Tyr 1068) decreased with increasing noscapine concentration, indicating that noscapine suppresses EGFR phosphorylation and that MG63 proliferation and migration are significantly reduced [53]. Furthermore, they concluded that noscapine suppresses the EGFR pathway by inhibiting the expression of cyclin D1 and CDK4/6 and prevents cell transfer from phase G1 to phase S, resulting in antiproliferative effects with induction of apoptosis on cells MG63 [53].

### 4.10. Effects of Noscapine on Nuclear Factor Kappa-Light-Chain-Enhancer of Activated B Cells (NF-*κ*B)

NF-*κ*B is a transcription factor that, by binding directly to DNA, regulates gene expression and the synthesis of various proteins involved in cellular processes such as survival, proliferation, invasion, and angiogenesis. This transcription factor is one of the essential regulators of proinflammatory gene expression, transcribing and synthesising cascades of cytokines and proinflammatory chemokines such as interleukin (IL)-1*β*, IL-6, and IL-8 and, consequently, causes inflammatory responses [132].

Altered NF-*κ*B activity is seen in different types of diseases, including stroke, severe epileptic seizures, brain damage, Alzheimer's, Parkinson's, gastric ulcer, Crohn's, Huntington's, and immune diseases such as psoriasis and cancers. Additionally, improper activation of NF-*κ*B in many malignancies, including glioblastoma, in which stem cells proliferate, causes tumour cells to invade surrounding tissues and resist radiation therapy [133].

Sung et al. observed that noscapine in human leukaemia and myeloma cells inhibited the expression of NF-*κ*B-controlled genes that are essential for the survival, proliferation, and angiogenesis of tumour cells [6]. Through IK*β*-kinase, noscapine, inhibits the activity of NF-*κ*B in malignant cells, leading to inhibition of phosphorylation and degradation of IK*β*-*α* [6]. Noscapine also blocks phosphorylation and nuclear translocation of p65 and inhibits NF-*κ*B reporter activity caused by various anticancer agents NF-*κ*B [6]. In addition, noscapine also inhibits NF-*κ*B downstream activity such as the cyclooxygenase-2 promoter [6, 134]. Noscapine has been shown to inhibit NF-*κ*B activity and tumour growth in animal models of triple-negative breast cancer, along with doxorubicin [36].

## 5. Conclusion

Noscapine is a herbal compound that has been used clinically as an antitussive since the 1950s. In recent years, various pharmacological properties of noscapine have been observed in cellular studies, including induction of apoptosis, decreased microtubule dynamics, inhibition of tumour cell growth, and inhibitory effects on NF-*κ*B, VEGF, and EGFR. In addition, noscapine has anti-inflammatory effects and significantly reduces the levels of proinflammatory factors such as IL-1*β*, IFN-*γ*, IL-6, TNF-*α*, and antioxidant effects by inhibiting NO and reducing ROS levels. Furthermore, noscapine inhibits the growth of cancer cells and prevents metastasis to other tissues. In addition, noscapine easily crosses the blood-brain barrier and exerts appropriate inhibitory effects on glioblastoma, which can be therapeutic. These therapeutic effects, along with low systemic toxicity, good oral bioavailability, and proper tumour targeting, have made noscapine a viable option for treating many inflammatory diseases and cancers. Furthermore, noscapine has been shown to have synergistic effects in cellular studies alongside conventional anticancer drugs.

## Figures and Tables

**Figure 1:** The possible signalling pathways modulated by noscapine.

**Figure 2:** Noscapine activates apoptosis in cancer cells by activating the C-jun N terminal kinase signalling pathway, inhibiting extracellular regulated kinase (ERK) signalling, and BCL-2 phosphorylation.

**Table 1:** Evaluation of the effect of noscapine on cancer cells along with other first-line drugs.

Noscapine	Anticancer drug	Type of cancer	Growth inhibition (%)	*In vivo or in vitro*	Ref.
150–550 mg/kg/day	Doxorubicin (1.5 mg/kg)	Triple negative breast cancer (TNBC)	39.4%–82.9% synergistic interaction between noscapine and doxorubicin	*In vitro* MDA-mb-231 and MDA-mb-468 cells	[36]
300 mg/kg/day	Gemcitabine (30 mg/kg)	Non-small-cell lung cancer (NSCLC)	82.9 ± 4.5 synergistic interaction between noscapine and gemcitabine	*In vitro* H460 tumors	[32]
225 mg/kg twice per day	TMZ (5 mg/kg)	Glioblastoma multiforme TMZ-resistant	Noscapine increased survival in the orthotopic *in vivo* xenograft model of TMZ-resistant glioma.	*In vitro* U251 and A172 cells	[30]
100 mg/kg/day	Docetaxel (0.4 *μ*M)	Triple negative breast cancer	30% increase in number of late apoptotic cells, synergistic interaction	*In vitro* MDA-mb-231 cells	[50]

**Table 2:** Anti-inflammatory effect, the antiapoptotic effects of noscapine.

Effects	Type of study	Model	Cancer type	Dose/Conc	Mechanism	Years	Ref
Inducing apoptosis	*In vivo*	Blocking CDH17 gene in colon cancer SW480 cells	Colon cancer cells	10 *µ*mol/L	↑Bax, ↓Bcl-2 and ↓Bcl-xL	2017	[135]
Antiproliferation	*In vitro* and *in vivo*		Triple negative breast cancer	100 mg/kg	Increase sensitivity to docetaxel	2017	[136]
Inducing apoptosis	*In vivo*	MCF7 cells	Breast cancer		Progression in G2/M transition	2021	[137]
Inducing apoptosis	*In vitro*	The expression of apoptotic genes significantly increased	Endometriosis	3 *μ*g/mL	Inhibiting angiogenesis and nitric oxide	2019	[138]
Antineuroinflammation	*In vivo*	Parkinson's disease		10 mg/kg	Enhancing the expression of mTOR and prevented apoptosis	2021	[139]
Inducing apoptosis	*In vitro* and *in vivo*	Human breast cancer cell lines MDA-MB-231 and MDA-MB-468	Breast cancer	50 mg/kg	Promoting effect on apoptosis-induced apoptosis in colon cancer cells via p53-dependent pathway reduces VEGF expression	2019	[140]
Anticancer	*In vivo*	LNCaP and PC-3 human prostate cancer cell lines	Human prostate cancer cell lines	50 *μ*M	↓Bcl-2-↑Bax, and ↑Bax/Bcl-2 ratio	2017	[141]
Inducing apoptosis -tubulins	*In vivo*	MCF-7 and MDA-mb-231	Breast cancer	1.35 ± 0.2 *μ*M	↑ROS ↓tubulin assembly	2020	[142]
Tubulin	*In situ*	STD-NMR		0.6 *μ*M	↓tubulin assembly	2020	[143]
Inhibition of p-glycoprotein	*In vivo*	Human breast adenocarcinoma cell line MCF7	Breast cancer	45.4 ± 6.5 *μ*M	↓P-gp function	2019	[102]
Inducing apoptosis	*In vivo*	The human colon cancer cell lines HT29 and LoVo	Colon cancer cells	75 *μ*M	↓PI3K/mTOR signalling-↓Warburg effect	2020	[56]
Inducing apoptosis	*In vivo*	U87 cells	Human glioblastoma cells	46.8 *µ*M	↑apoptosis	2019	[144]
Antiangiogenic	*In vivo*	Human umbilical vein endothelial cells	Endothelial cells	11.87 *μ*M for Cl-noscapine, 6.9 *μ*M for Br-noscapine, and 6.79 *μ*M for folate-noscapine	Antiangiogenesis activity	2018	[116]

^*∗*^STD-NMR: Saturation transfer difference (STD) Nuclear Magnetic Resonance (NMR).

## Data Availability

No data were used to support this study.

## Abbreviations

ACE: Angiotensin-converting enzyme
ADP ribose: Adenosine diphosphate ribose
AIF: Apoptotic inducing factor
BBB: Blood-brain barrier
BCL-2: Antiapoptotic downregulation
bFGF: Basal fibroblast growth factor
BK: Bradykinin
COX-2: Cyclooxygenase-2
cGMP: Cyclic guanosine monophosphate
C-JNK: C-jun N terminal kinase
Cys: Cysteine
DOX: Doxorubicin
EGFR: Epidermal growth factor receptor
ERK: Extracellular regulated kinase
FDA: Food and Drug Administration
GBM: Glioblastomas
GSH: Glutathione
GluT1: Glucose transporter
GRB2: Growth factor receptor-bound protein 2
HIF-1: Hypoxia-inducible factor-1
HUVECS: Human umbilical vein endothelial cells
HK2: Hexokinase 2
IL-1*β*: Interleukin 1 beta
IL-6: Interleukin-6
IL-8: Interleukin-8
IFN-*γ*: Interferon-gamma
IKK: IK*β*-kinase
KKS: Kallikrein-kinin system
LDHB: Lactate dehydrogenase B
MAPK: Mitogen-activated protein kinase
MCP1: Monocyte chemoattractant protein 1
MMP: Matrix metalloproteinase
mg/kg: Milligram/kilogram
MGMT: Methylguanine methyltransferase
NADPH: Nicotinamide adenine dinucleotide phosphate
NCI: National Cancer Institute
NO: Nitric oxide
NPN: N-Propargyl noscapine
NMDA: *N*-Methyl-D-aspartic acid
NRFs: Nuclear transcription factor
PTEN: Phosphatase and tensin homolog
PIP3: Phosphoinositide 3
PI3K: Phosphoinositol tri-kinase
P-gp: P-glycoprotein
PPARs: Peroxisome proliferators
PKM2: Pyruvate kinase M2
ROS: Reactive oxygen species
TLR: Toll-like receptor
TNF-*α*: Tumor necrosis factor-alfa
TNBC: Triple-negative breast cancer
VEGF: Vascular endothelial growth factor
3-MA: 3-Methyladenine.
